# Empowerment assessment and influential factors among patients with type 2 diabetes

**DOI:** 10.1186/2251-6581-12-6

**Published:** 2013-01-19

**Authors:** Azar Tol, Abdolvahab Baghbanian, Bahram Mohebbi, Davoud Shojaeizadeh, Kamal Azam, Sima Esmaeeli Shahmirzadi, Abolghasem Asfia

**Affiliations:** 1 Department of Health Education and Promotion, School of Public Health, Tehran University of Medical Sciences, Tehran, Iran; 2 Health Promotion Research Center, Zahedan University of Medical Sciences, Zahedan, Iran; 3 School of Medicine, Tehran University of Medical Sciences, Tehran, Iran; 4 Department of Biostatistics, School of Public Health, Tehran University of Medical Sciences, Tehran, Iran; 5 Department of Education and Promotion, School of Public Health, Tehran University of Medical Sciences, 4th Floor, School of Public Health, Pour Sina Ave, Tehran, Iran

**Keywords:** Empowerment, Type 2 diabetes, Diabetic patients

## Abstract

**Background:**

Diabetic patients need high awareness of disease prevention to adopt self-management behaviors in their daily life. Central to this activity is patients’ empowerment. Current study was conducted to assess empowerment score and its related factors among type 2 diabetic patients.

**Method:**

A cross-sectional study carried out over a period of nine months during 2010–2011. All patients with a diagnosis of type 2 diabetes including those referring to four hospitals affiliated with Tehran University of Medical Sciences were recruited. A total of 688 diabetic patients were identified who met the inclusion criteria and were all included in the study. Patients’ empowerment was measured by Diabetes Empowerment Scale reflecting three dimensions including managing psychosocial aspect of diabetes, assessing dissatisfaction and readiness to change and Setting and achieving diabetes goal. Collected data was analysed using SPSS software version 11.5.

**Results:**

As total, 688 were available for analysis, ranging from 37–81 years old with mean of 54.41 years (SD = 8.22). The Mean duration of the disease was approximately 6.67 years (SD = 4.58). Dimensions of ‘managing the psychosocial aspect of diabetes’, ‘assessing dissatisfaction and readiness to change’ and ‘setting and achieving diabetes goal’ were all measured and scored for each patient. The mean score for each domain was 25.75 ± 5.55, 24.78 ± 7.54, 27.63 ± 7.90, respectively. Data analysis revealed a statistically significant reverse relationship between age and ‘assessing dissatisfaction and readiness to change’ and ‘setting and achieving diabetes goal’. In addition, disease duration had a statistically significant reverse relationship with ‘assessing dissatisfaction and readiness to change’.

**Conclusion:**

Patients with type 2 diabetes have the potential to be empowered to manage their chronic disease if they are actively informed and educated.

## Introduction

Type 2 diabetes is a metabolic illness, and an increasingly prevalent condition around the world whereby the human body is unable to make enough or properly use insulin [1]. World Health Organization (WHO) estimates that diabetes is becoming a global epidemic of the 21^st^ century, and that over 70% of known cases of diabetes belong to developing countries [2]. In Iran the prevalence of disease is reported to be between 2–10% among adults [3]. The Iranian Ministry of Health and Medical Education (MOHME) has reported a prevalence of 2.3% [4] in Tehran, only.

Neither the curative and medical approaches towards dealing with patients and disease nor the compliance/adherence model of care is effective in diabetes care [5]. Diabetic patients demand long-term and continuous self-care, self- management and preventive care behaviors. They play a fundamental role in the process of treatment [6-10]. This reflects that health cannot merely be achieved outside the individual’s own control by professionals but necessitate the patients’ active participation in health care [11].

An innovative approach and a real paradigm shift is required to recognize that patients are in control of and responsible for the daily self-management of diabetes [6]. This new approach, based on the issue of ‘empowerment ’, is more valid about day to day activities in type 2 diabetic patients [12]. It is based on the three fundamental aspects of chronic illness care: choices, control, and consequences – which make it much more applicable for disease prevention [13,14]. Cooper and et al. (2008) noted that empowerment of diabetic patients certainly would help them adopt an appropriate healthy behavior, and improve self- management practices [15].

Generally, ‘empowerment is a practice which people achieve greater control over their own decisions and practices affecting their health’ (WHO, 1998). As a positive concept and outcome empowerment is regarded as recourses beside to defects, and helps patients to identify and learn to solve their own problems. As a process, it facilitates health care process and interactions to overcome patients’ problems [6]. While empowerment improves the ability and innate capacity of patients to better cope with their disease, it is a vital concept of promoting patients’ overall well-being [16].

Diabetic patients must take responsibility for their care plan and make appropriate decisions on their daily activities [17,18].

This study aims to assess the empowerment score and its related factors among type 2 diabetic patients referring to four hospitals affiliated with Tehran University of Medical Sciences. The study has the potential to increase our understanding about patient and family empowerment, and can help policy-makers make appropriate and timely decisions.

## Methods

### Study design and participants

A cross-sectional study was carried out over a period of nine months during 2010–2011 in Tehran, Iran. Using continuous sampling method, 688 type-2 diabetes patients, who had referred to four teaching hospitals (including Imam Khomeini, Shariati, Amir-Alam, Baharlou) affiliated with Tehran University of Medical Sciences, were selected to participate in the study. Patients were eligible to participate if they had at least 35 years old, as well as type-2 diabetes being diagnosed for a minimum of one year. All patients were informed about the aim of study. No patient was forced or obliged to participate in the study. Consent form was obtained from each patient.

### Instrument

Data gathering was performed through a self-reporting questionnaire. It consisted of two sections: First section was related to socio-demographic information and the second part included a 28-item Diabetes Empowerment Scale (DES-28) which developed by the University of Michigan Diabetes Research and Training Center [19,20].The DES is a self-report scale and contains three subscales including a) managing the psychosocial aspects of diabetes with 9 items, b) assessing dissatisfaction and readiness to change with 9 items, and c) setting and achieving goals with 10 items. Each scale item has five response-categories ranging from 1 to 5 (1 = strongly disagree, 2 = somewhat disagree, 3 = Neutral, 4 = somewhat agree, 5 = strongly agree). Accordingly, the minimum and maximum scale values were 28 and 140, respectively. The overall scores represented the overall DES and higher scores indicated a better DES. The validity and reliability of the Persian version of the scale was tested by Tol et al. The psychometric analysis was used to evaluate the reliability and validity of the scale including its three subscales as follows: managing the psychosocial aspects of diabetes (α = 0.94), assessing dissatisfaction and readiness to change (α = 0.96), and setting and achieving diabetes goals (α = 0.96).Interclass correlation coefficient and test-retest reliability were used for stability analysis and was satisfactory (p < 0.001). Criterion validity between DES score and metabolic control (HbA1c) patients with type 2 diabetes was approved (p < 0.001) [21].

### Statistical analysis

Data analysis was conducted using SPSS software version 11.5. Descriptive statistics were used for all variables. Non-parametric test (Mann–Whitney U) was also used for variables with non-normal distributions. In addition, Pearson’s and Spearman’s correlation coefficients were used to assess the relationship between numeric variables. The significance level was set at p < 0.05.

## Results

Participants were aged between 37 to 81 years old with a mean of 54.41 years (SD = 8.22). Almost 47.5% was male, 86.6% was married, and 44.9% had diploma and higher levels of education. The mean duration of the disease was 6.67 years (SD = 4.58) (Table 1). Using Diabetes Empowerment Scale, three conceptual domains of ‘managing the psychosocial aspect of diabetes’, ‘assessing dissatisfaction and readiness to change’ and ‘setting and achieving diabetes goal’ were all measured and scored for each patient. The mean score of each domain was (25.75 ± 5.55), (24.78 ± 7.54), (27.63 ± 7.90) respectively. The dimension of the ‘setting and achieving diabetes goal’ was reported to be the most important domain in measuring Self-care and empowerment in diabetes care.

**Table 1:** Demographic and clinical characteristics of patients with diabetes

**Variables**	**(%) number**, **N = 688**
**Gender**	
female	(52.5) 361
male	(47.5) 327
**Educational level**	
Illiterate	(14.2) 98
Up to diploma	(78.5) 540
higher than diploma	(7.3) 50
**Marital status**	
Unmarried	(13.4)92
married	(86.6)596
**Disease duration**	
<5 years	(51.7) 356
5-10 years	(30.6) 210
> 10 years	(17.7) 122
**History of diabetes**	
Yes	(69.8) 480
No	(30.2) 208

Pearson’s correlation coefficient showed a statistically significant reverse relationship between patients’ age and dimensions of ‘assessing dissatisfaction and readiness to change’ (r = −0.105, p = 0.006) and ‘setting and achieving diabetes goal’(r = −0.101, p = 0.008). Furthermore, the duration of disease had a statistically significant reverse relationship with ‘assessing dissatisfaction and readiness to change’ (r = − 0.1, p = 0.009). Often, with increasing age among diabetes patients, their empowerment score would decrease in terms of the dimensions of ’assessing dissatisfaction and readiness to change’ and ‘setting and achieving diabetes goal’. Also, with increasing the duration of disease, the score for ‘assessment of dissatisfaction and readiness to change’ would decrease.

Furthermore, Spearman’s correlation coefficient showed that the level of education had a statistically significant direct relationship with ‘managing the psychosocial aspect of diabetes’ (r = 0.078, p = 0.04), ‘assessing dissatisfaction and readiness to change’(r = 0.076, p = 0.04) and ‘setting and achieving diabetes goal’(r = 0.09, p = 0.01) (Table 2). This finding implies that with increasing education, all dimensions of the empowerment concept would increase. The total scores for empowerment had a significant relationship with the patients’ level of education (F = 3.70, P = 0.01).

**Table 2:** The correlation between empowerment components and demographic variables

**Variables**	**Managing psychosocial aspects of diabetes**		**Assessing dissatisfactionand readiness to change**		**Setting and achieving diabetes goals**	
	**Coefficient correlation**	**P**-**value**	**Coefficient correlation**	**P**-**value**	**Correlation coefficient**	**P**-**value**
**Age**	−0.036	>0.05	−0.105*	0.006	−0.101*	0.008
**Level of Education**	0.078*	0.04	0.076*	0.04	0.095*	0.01
**Disease duration**	0.010	>0.05	−0.1*	0.009	−0.046	>0.05

## Discussion

The current study was conducted to assess the empowerment score and its related factors among patients with type 2 diabetes. According to the results, ‘setting and achieving diabetes goal’ was considered to be the most important factor in measuring diabetes self-empowerment. The overall score of empowerment had a significant relationship with the patients’ level of education.

The main purpose regarding the management of chronic diseases such as type 2 diabetes is to encourage patients to take greater responsibility for their care, and to perform self – management practices [21].

Healthcare professionals and academics have introduced self-empowerment as an important factor in managing chronic diseases. When it comes to diabetes management, empowerment involves an innovative approach that attempts to improve the ability of patients to actively understand and influence their own daily living activities and health status (Reference). This approach helps diabetic patients make rigorous decisions about their own care plan, to better overcome their disease [15,22].

Effective empowerment of patients is not achieved unless patients obtain the necessary knowledge and skills, and are educated about their own health status [12].

Current study findings revealed that the dimension of ‘setting and achieving diabetes goals’ has gained the highest mean score. It is probable that years of living with diabetes can affect patients in adopting healthy practices through empowerment. This finding can be explained by the fact that younger patients with diabetes seek more information, and are more sensitive to diabetes aspects relative to older patients. In contrast, with increasing age and duration of the disease, diabetes patients show low readiness to change their situation. These findings are in contrast with Liu’s study that showed that with increasing age, the patients’ empowerment score has increased [17].

In addition, the study findings revealed a significant relationship with patients’ level of education: higher levels of education provide better empowerment scores. This finding represents that patients with type 2 diabetes are able to self-empower and self-manage their disease if they are enthusiastically informed and educated. Accordingly, the patients’ compatibility with disease would increase which is the result of relationship between patients’ self- efficacy, self- esteem and self-empowerment, as has been reported by Alhani elsewhere [23]. Alhani argued that self-esteem improves self-control and leads to enhancing self-efficacy that is along with an increase in empowerment level.

Empowered patients are capable to control their daily self-care decisions that diabetes requires [10] as has been reported by Anderson where the author shows any improvement in patients’ empowerment would result in managing and controlling diabetes [9,10].

Patient empowerment is also considered as an intervention strategy that enables policy-makers perform accurate health promotion interventions [24] as it creates an active interaction between providers and their patients [25]. This mutual relationship can facilitate the patient empowerment – being a key component of self-management adoption [22], and is helpful to improve trust between patients and providers [26].

Patients who are actively collaborating in the decision-making process are better able to achieve the outcomes they identify as important to them.

Focusing on appropriate knowledge, skills and practices, dynamic participation of patients in decision-making process would lead to achieving better outcomes about their disease. This allows patients to adopt healthy practices as the main pathway to diabetic empowerment [27-30]. As well, this fact should be considered that beside of named factors, assessing diabetes distress and attitude towards diabetes with appropriate tools in order to achieve better adherence to diabetes care plan can be useful [31,32].

## Competing interests

The authors declare that they have no competing interests.

## Authors’ contributions

AT carried out the implementation and data collection of the study, AB Participated in the sequence alignment and drafted the manuscript, BM made medical consultation for the study, DSH help start the study, KA participated in analyzing statistics of the manuscript, SSSH help data gathering and participation to implementation of study, AA participated in planning the study and help in discussion of the manuscript, All authors read and approved the final manuscript.
